The article "KDOAM-25 Overcomes Resistance to MEK Inhibitors by Targeting KDM5B in Uveal Melanoma" was retracted in 2023. Reasons: unreliable results or conclusions; concerns about the data; concerns about the peer review; concerns about the citations.

# KDOAM-25 Overcomes Resistance to MEK Inhibitors by Targeting KDM5B in Uveal Melanoma

**DOI:** 10.1155/2022/1556485

**Published:** 2022-09-28

**Authors:** Hongjun Zhang, Xiangnan Liu, Yong'an Chen, Rui Xu, Shengli He

**Affiliations:** ^1^Department of Ophthalmology, Minhang Hospital, Fudan University, Shanghai, China; ^2^Department of Ophthalmology, Changhai Hospital Affiliated to Naval Medical University, Shanghai, China; ^3^Department of Oncology, Naval Medical Center of Chinese People's Liberation Army, Naval Military Medical University, Shanghai, China; ^4^Division of Rheumatology, Huashan Hospital, Fudan University, Shanghai, China; ^5^Department of Hepatobiliary-pancreatic and Integrative Oncology, Minhang Branch, Fudan University Shanghai Cancer Center, 106 Ruili Road, Minhang District, Shanghai, China

## Abstract

**Background:**

Uveal Melanoma (UM) is a potentially lethal cancer, and epigenetics may participate in the regulation of MEK resistance. This study is aimed at targeting the epigenetic kinase to overcome the resistance to MEK inhibitor.

**Method:**

We developed the 92.1 and OMM1 MEK-inhibitor resistant cell lines by culturing them in the trametinib (Tra) mixed medium. We utilized CCK8 analysis for detecting the viability of the cell. Western blot was used to determine the ERK1/2 and Akt phosphorylation. Small compound library screening assays were carried out by CCK8 analysis. To test the apoptosis, we employed flow cytometric analysis with Annexin-V/PI. Western blot and CCK8 were used to explore the epigenetic regulation of KDM5B in MEK-resistance cell lines. To knock out the expression level of KDM5B, we used the CRISPR/Cas9 by lentivirus delivering well-validated shRNAs in pLKO.1 vector. The directly binding affinity of KDOAM-25 to KDM5B was determined by drug affinity responsive target stability (DARTS) and microscale thermophoresis (MST).

**Results:**

The phosphorylation of ERK1/2 and Akt (T308) was inhibited in OMM1 cell lines. However, inhibition of Tra was abolished in OMM1-R cell lines. From a compound screening assay, we identified that KDOAM-25 robustly inhibited the viability and colony formation of MEK-resistance cell lines. Furthermore, KDOAM-25 significantly promoted cell death in OMM1-R cells. H3K4me3 (tri-methylation of lysine 4 on histone H3) and H3K27ac (acetyl of lysine 27 on histone H3) were both upregulated in OMM1-R cells. Tra significantly inhibited the expression of KDM5B in OMM1-P cells. However, the effect on KDM5B was abolished in OMM1-R cells. Knockdown of KDM5B robustly suppressed the cell viability in OMM1-R cells. KDOAM-25 directly interacted with KDM5B.

**Conclusion:**

KDOAM-25 inhibited the viability and colony formation and promoted cell death of MEK-resistance cell lines through H3K4me3 and H3K27ac, indicating that KDOAM-25 may be a potential therapeutic agent for MEK resistance in UM patients.

## 1. Introduction

Uveal melanoma (UM) is a potentially lethal cancer with an annual incidence of 0.002‰ to 0.008‰ [1], but factors determining the unfavorable course of this disease are still unknown. The clinical goal of UM treatment is to control tumor growth and prevent tumor metastasis. Despite the primary tumor being already local control, overall survival (about 80% at 5 years) has not improved significantly over the past 40 years. About 50% of patients develop metastatic UM (mUM), with a median survival of fewer than 12 months. The study found that 90% of metastases involved the liver, with the average survival time of untreated patients as only about 2 months and the average survival time of treated patients as about 6 months [2, 3]. At present, there is no standard treatment for mUM. So it is important to investigate the mechanism of UM to address the potential therapeutic approach.

Given that UM is highly resistant to chemotherapy and immunotherapy-based approaches, therapeutic compounds specifically targeting dysregulated oncogene molecular pathways could serve as attractive alternatives [2–4]. Targeted therapy has been proved to have great beneficial in cancers with specific targeting [5], such as the good prognosis in endothelial growth factor receptor- (EGFR-) mutated non-small-cell lung cancer (NSCLC) after treatment with EGFR inhibitors, breast cancer gene- (BRCA-) mutated ovarian cancer with poly-ADP- (adenosine diphosphate-) ribose polymerase (PARP) inhibitors, and treatment of BRAF-mutated cutaneous melanoma, as well as NSCLC with BRAF inhibitors or MEK inhibitors [6–9]. Approximately 90% of UM patients have mutually exclusive mutations in the two homologous G protein alpha subunits, GNAQ and GNA11, which are early events and drivers of UM development, leading to constitutive activation of the mitogen-activated protein kinase (MAPK)/ERK pathway [10].

Activation of the MAPK/ERK pathway is a well-described oncogenic event involving a cascade of consecutive activation of RAS, RAF, and MEK. And the inactivation of ERK leads to cell proliferation and survival [11]. Inhibition of MEK has also been investigated as a promising therapy in UM [12]. Although the use of MEK inhibitors has a good clinical effect, it may cause resistance to MEK inhibitors in patients. Therefore, it is urgent to determine the mechanism of MEK inhibitor resistance in UM.

Epigenetic modification is the study of heritable changes in gene function that does not involve changes in the DNA sequence, including DNA methylation, histone modifications, noncoding RNA, and chromosome stability [13]. Among the diverse histone modifications, methylated lysine is the best-understood marker of histone code, as specific methylated lysine match well with gene expression states. In general, H3K4me2/3 residues indicate the transcriptional start site of active transcriptional genes, whereas demethylation of H3K4 is related to transcriptional repression [14]. KDM5B (Lysine Demethylase 5B), a histone-specific demethylase containing 1544 amino acids, shows a restricted expression pattern in adult tissues and is primarily present in the testis and brain [14]. Studies have shown increased KDM5B levels in a variety of human cancers [15]. And in recent studies, KDM5B is considered a transcriptional repressor and associated with tumor growth, angiogenesis, invasion, metastasis, and tumor-associated chemoresistance. However, the mechanism of KDM5B in the MEK-inhibitor resistance patients in UM remains unclear.

In the present study, a high-throughput screening assay was performed to identify the small compound KDOAM-25, which directly binds to KDM5B and robustly overcomes the MEK-inhibitor resistance in UM. This will throw new light on the treatment of UK.

## 2. Materials and Methods

### 2.1. Generation of MEK Inhibitor-Resistant Cell Lines

We cultured the 92.1 and OMM1 parental cells in the RPMI-1640 medium which contains fetal bovine serum (10%). Then, we seeded the cells (5,000 cells per well) into 96-well plates for 24 h. We cultured the cells in the Tra-supplemented medium, and most cells are dead. The survived cells are continually feeding in the Tra-supplemented medium. In the interval of 2 days, we resuspended the cells in fresh medium supplemented with Tra. Then, the survived cells were collected and CCK8 analysis was used to detect cell viability. We doubled the Tra dose for collecting more than 30-fold drug-resistant cells in comparison with their original parent cells when cell viability was more than 90%.

### 2.2. Western Blot

OMM1 parental cells and resistant cells were seeded into 6-well plates and harvested after cultured for 12 h. Cells were then collected to the Cell lysis buffer (CST, USA) supplemented with protease and phosphatase inhibitor cocktail (Roche, Switzerland) after being treated with Tra (5 *μ*M). The lysed protein was loaded on a 10% polyacrylamide gel for SDS-PAGE, then moved into the PVDF membrane at 270 mA for 90 min. The membrane was blocked in 5% fat-free milk for 1 h at room temperature and incubated with the indicated primary antibodies at 4°C overnight: p-ERK (#9101), p-Akt (#4060), and *β*-actin (#4967) were from Cell Signaling Technology; H3K4me3 (ab8580) and H3K27ac (ab4279) were from Abcam; KDM5B (MA5-31785) is from Thermo Fisher. The membrane was washed three times by using the TBST and probed with secondary antibodies which is collected from Proteintech, China. Finally, we used the imaging system (Tanon, Shanghai, China) for collecting substantial images.

### 2.3. CRISPR/Cas9-Mediated KDM5B Knockdown

We knocked down the KDM5B by retroviruses delivering well-validated shRNAs in the MSCV-LMP vector. We cloned the gRNAs targeting KDM5B or GFP into a vector encoding espCas9. The gRNA sequences targeting KDM5B are 5′-ATGCCAGTCCTCGGCTATGGG-3′ and 5′-GCCCGGTCTGAACCCAGCTGG-3′. According to the guidelines of the manufacturer (Thermo Fisher, USA) for using PEI transfection reagent, we generated and collected retroviruses by cotransfection of HEK293FT cells which contain the packaging vectors PCL-ECO (Addgene). After transfection of 48-72 h, we harvested the retrovirus supernatants and centrifuged it at a speed of 2500 rpm for 10 min at room temperature. We removed the cells debris by filtering the supernatant with a filter (0.45 *μ*m). We infected the cells by using 8 *μ*g/mL Polybrene (Chemicon, Temecula, CA, USA) and the virus stock. After 48-72 h, 0.5 *μ*g/mL puromycin (Invitrogen, USA) was used for selecting the infected cells. The survived cells were cultured continually to establish stable cell lines. The cell clones were selected to detect the knockdown efficiency by Western blot using KDM5B antibodies.

### 2.4. CCK8 Assay

We assessed the viability of 92.1 and OMM1 parental and resistant cells by using the CCK8 assay (TopSCIENCE, China) as guided by the manufacturer company. 92.1 and OMM1 parental and OMM-resistant cells were placed into 96-well plates with 2 × 10^4^ cells/well. After cells were plated, we incubated the cells in a Tra-supplemented medium with indicated concentrations. After 72 h, the cells were added with 10 *μ*L of CCK8 stock solution and incubated the supplied cells for 2-4 h at 37°C optimum temperature. We measured the OD value at 450 nm.

### 2.5. Flow Cytometric Analysis of Apoptotic Cells

The parental OMM1 and OMM1-respective resistant cells were mixed with KDOAM-25 (5 *μ*M) for 24 h and washed cell with PBS two times. Cells were stained with Annexin V-FITC kit (Yeasen, China) according to the manufacturer. Briefly, cells were resuspended by the binding buffer and stained with Annexin V and PI for 15 min at room temperature in the binding buffer. We conducted the flow cytometry analyses on Fortessa X20 (BD Biosciences) system. We analyzed the generated data by using FlowJo V10 software.

### 2.6. Protein Labeling and Microscale Thermophoresis (MST) Binding Assay

His_6_-MBP-KDM5B was labeled with RED-tris-NTA 2nd Generation using the MONOLITH NT.115. The binding of inhibitors to KDM5B was evaluated using MST. Ligands (49 nM–150 *μ*M) were incubated with 100 *μ*L 100 nM RED-tris-NTA 2nd Generation dye in the dark for 30 min in assay buffer (20 mM HEPES at pH 7.4, 150 mM NaCl, 0.05% Tween 20). The sample was loaded into NanoTemper Monolith NT.115 glass capillaries, and MST was carried out using 40% MST power. *K*_*d*_ values were calculated using the mass action equation and NanoTemper software.

### 2.7. Drug Affinity Responsive Target Stability (DARTS)

DARTS was performed according to a modified published protocol. Purified HIS-KDM5B proteins were diluted by 100 mM phosphate buffer, pH 7.4 to a final concentration of 0.04 *μ*g *μ*L^−1^. The proteins were treated with Tra (final concentration of 50 *μ*M; dissolved in DMSO) for 1 h, and equal amounts of DMSO were added to the solutions, which served as control samples. Pronase (Roche) was dissolved in TNC buffer (50 mM Tris-Cl, 50 mM NaCl, 10 mM CaCl_2_, pH 7.5). The 0.05 *μ*g of pronase was added to the protein solution (100 *μ*L) and incubated in the mixed solution for 1 h at 37°C temperature. We stopped the pronase reaction by adding 5× SDS loading buffer. Then, the samples were boiled at 95°C for 15 min and loaded on SDS-PAGE gels. After SDS-PAGE, gels were used for western blot analysis. A total of 30 *μ*g of protein extract was separated on 10% SDS-PAGE gels and transferred to nitrocellulose membranes. For the dimerization studies, cell lysates were analyzed on native (nondenaturing) gels.

### 2.8. Statistical Analysis

All statistical analyses were performed utilizing GraphPad Prism 7 (GraphPad Software). Statistical significance was calculated using unpaired Student's *t*-tests to compare the means of two groups, one-way analysis of variance (ANOVA) or two-way ANOVA, to compare the means of three or more groups.

## 3. Results

### 3.1. Evolution of MEK Inhibitor Resistance in UM Cells

To explore the mechanism of drug resistance in UM cells, we generated the resistant cells using 92.1 and OMM1 UM cell lines, which are sensitive to the Tra. The viability data showed that parental 92.1 cell lines (92.1-P) were killed being treated with Tra in a dose- and time-dependent manner (Figures 1(a) and 1(b)). Similar results were observed in OMM1 cell lines (OMM1-P) (Figures 1(c) and 1(d)). The phosphorylation of ERK1/2, the downstream signal molecule of the MEK signal pathway, was upregulated in the OMM1-R cell compared with the OMM1-P cell (Figures 1(e) and 1(f)). Given the critical role of mTOR in MEK inhibition UM cells, the activation of the p-Akt was detected, which is a key signal in the mTOR pathway. The data showed that the phosphorylation of Akt was upregulated in OMM1-R cells compared with OMM1-P cells (Figures 1(g) and 1(h)). Thus, we generated MEK inhibitor-resistant cells in 92.1 and OMM1 UM cells.

### 3.2. KDOAM-25 Overcomes the MEK Resistance in MEK Inhibitor-Resistant UM Cells

To investigate whether there is a candidate target epigenetic modification kinase in MEK inhibitor-resistant UM cells, a small molecule compound library was conducted, which targets epigenetic molecules, and the viability after treating the 92.1-R cells with the compounds was analyzed. The data showed that KDOAM-25 significantly suppressed the viability of 92.1-R cells (Figure 2(a)). Furthermore, a lower concentration of KDOAM-25 abolished the colony formation capability of 92.1-R cells but showed no effect on 92.1-P cells (Figure 2(b)). Similarly, the viability of 92.1-R was significantly suppressed by KDOAM-25 (Figure 2(c)). To further confirm the effect of KDOAM-25 on the MEK-resistant cells, the apoptosis of the cells were detected by flow cytometric analysis. We found an increased percentage of apoptotic cells (Annexin-V^+^) after treatment with KDOAM-25 (Figures 2(d) and 2(e)). Therefore, we identified that KDOAM-25 could overcome the resistance of MEK in UM cells.

### 3.3. KDOAM-25 Overcomes Resistance to MEK Inhibitor by Targeting KDM5B in Uveal Melanoma

To investigate the mechanism of KDOAM-25 in the UM cells, we hypothesize that epigenetic modification may have a role in the MEK resistance. Firstly, the H3K4me3 (tri-methylation of lysine 4 on histone H3) and H3K27ac (acetyl of lysine 27 on histone H3) were found upregulated in OMM1-R cells (Figures 3(a) and 3(b)). Tra significantly inhibited the expression of KDM5B in OMM1-P cells (Figures 3(c) and 3(d)). However, the inhibition effect on KDM5B was abolished in OMM1-R cells (Figures 3(c) and 3(d)). To further investigate the role of KDM5B in MEK inhibitor cells, we knocked down the expression of KDM5B in OMM1-R cells, the knockdown efficiency was confirmed by western blot analysis (Figures 3(e) and 3(f)). Knockdown of KDM5B robustly suppressed the cell viability in OMM1-R cells (Figure 3(g)). Together, KDOAM-25 overcomes resistance to the MEK inhibitor by targeting KDM5B in UM.

### 3.4. KDOAM-25 Directly Binds to KDM5B

To further investigate the relationship between KDOAM-25 with KDM5B, we carried out the drug affinity responsive target stability (DARTS) assay, which is based on the altered protease susceptibility of target proteins upon drug binding. DARTS assay showed that when treated with KDOAM-25, KDM5B showed a differential pronase-dependent proteolysis pattern (Figures 4(a) and 4(b)). Furthermore, we used microscale thermophoresis (MST) to quantify the direct interaction between KDOAM-25 and KDM5B. The MST binding assay revealed that KDOAM-25 binds to KDM5B with a dissociation constant of 487.75 nM (Figure 4(c)). Thus, KDOAM-25 directly interacted with KDM5B.

## 4. Discussion

Patients who have completed standard chemotherapy due to drug resistance are an important issue. MEK inhibitor combinations have been approved for use in various cancers by the FDA [16]. However, cancer cells escaped from the function of MEK-inhibitor. Conceptually, our finding provides an example of applying “compound-mediated epigenetic silencing” to overcome the resistance of MEK-inhibitor. We found that the small molecule compound KDOAM-25 overcomes the resistance of MEK-inhibitor by directly binding to KDM5B. KDM5B acts as an oncogene; it is attractive to discover the potential KDM5B inhibitor for clinical use.

Epigenetic modification plays an essential role in cancer initiation and progression [13, 17]. Disruption of the epigenetic process leads to the altered gene function and malignant cellular transformation [18, 19]. Global changes in the epigenetic landscape are a hallmark of cancer. The epigenetic modification in cancer is characterized by global changes. DNA methylation, which was the first epigenetic alteration, plays an essential role in tumorigenesis. DNA hypomethylation may lead to genome instability of oncogenes, while loss of DNA methylation led to aberrant activation of oncogenes. The changes result in the dysregulation of gene expression, thus leading to cancer progression. DNA hypomethylation of a tumor suppressor is a common event in tumorigenesis. In addition, p16^INK4a^, also called cyclin-dependent kinase inhibitor 2A, plays an essential role in patients with progressing UM [20]. Histone modification, such as histone acetylation or methylation, methylation, phosphorylation, or ubiquitination, is found in various types of cancer [21–24]. Also, in a previous study, the histone methyltransferase EZH2, which is a component of the polycomb repressive complex 2, is involved in CIITA-PIV chromatin regulation in UM patients [20]. And in a recent study, the CUX2/KDM5B/SOX17 axis affects the occurrence and development of breast cancer [25]. The H3K4 trimethylation of transcription factor HES1 in UM cells caused overexpression of HES1, resulting in UM metastatic capacity.

Inhibition of MAPK has been proposed as an efficient means to enhance the clinical efficiency with the constitutive activation of the MAPK/ERK pathway. And it also has been investigated in UM [26, 27]. MEK inhibition promotes the percentage of CD8^+^ T cells in the tumor microenvironment and protects cells from death in the colon cancer model. However, MEK inhibition therapy often shows resistance in clinical uses. To determine the potential pathways that participated in the mechanism of resistance to MEK inhibitor, we collected and analyzed the clinical data from TCGA in UM patients. The inhibition of KDM5B correlates with longer survival and benefits. A previous study demonstrated that deficiency of KDM5B enhances the antitumor immunity and improves the survival after anti-PD-1 treatment [28]. Our study supports the application of the KDM5B inhibitor in clinical therapy in UM.

The KDM5 enzymes play essential roles in normal development and pathological conditions [15]. KDM5A is associated with the control of cell proliferation and differentiation in various cancer. KDM5B, also called PLU-1/JARID1B, is responsible for erasing the H3K4me2/3 activation marker [14]. Amounting evidence has demonstrated the oncogenic function of KDM5B in inhibiting the expression of tumor suppressors [15]. The di/tri-methylation of H3K4 represents the activation of the transcription genes at the transcription initiation sites; demethylation of H3K4 is marked by transcription gene repression, which may regulate cell proliferation, differentiation, and stem cell self-renewal. Thus, targeting KDM5B is an attractive approach for cancer therapy [15]. KDOAM-25 is a novel and selective KDM5B inhibitor, which has been demonstrated to inhibit KDM5B and used to investigate H3K4 methylation biology [29]. However, the role of KDOAM-25 in UM remains largely unknown. Our study showed that KDOAM-25 overcomes the MEK resistance by targeting KDM5B in UM. In a recent study, KDM5B regulates the PTEN/PI3K/Akt pathway to increase sorafenib resistance in hepatocellular carcinoma [30]. Also, one possible explanation resides in the fact that the small compound KDOAM-25 may eventually be inhibiting the expression of KDM5B, resulting in the upregulation of H3K4me3 and H3K27ac, consequently leading to the sensitivity to the MEK inhibitor in UM.

Still, there are some limitations of our study. We should not only verify the mechanism in our in vitro system but also in the in vivo system. So the animal model of melanoma should provide and use KDOAM-25 to investigate the effect on tumor growth and KDM5B expression in tumor cells from mice.

Collectively, our data showed by using a compound screening assay, we identified that KDOAM-25 robustly inhibited the viability and colony formation of MEK-resistance cell lines. Furthermore, KDOAM-25 significantly promoted cell death in OMM1-R cells. H3K4me3 (tri-methylation of lysine 4 on histone H3) and H3K27ac (acetyl of lysine 27 on histone H3) were both upregulated in OMM1-R cells. Tra significantly inhibited the expression of KDM5B in OMM1-P cells. However, the effect on KDM5B was abolished in OMM1-R cells. Knockdown of KDM5B robustly suppressed the cell viability in OMM1-R cells. KDOAM-25 directly interacted with KDM5B. In conclusion, KDOAM-25 inhibited the viability and colony formation and promoted cell death of MEK-resistant cell lines through H3K4me3 and H3K27ac, indicating that KDOAM-25 may be a potential therapeutic agent for MEK resistance in UM patients.

## Figures and Tables

**Figure 1:** Evolution of MEK inhibitor-resistant in UM cells. The CCK8 assay of cell viability in 92.1 parental (92.1-P) or 92.1-resistant (92.1-R) cells treated with Tra with indicated concentrations for 72 h (a) or indicated times with Tra (5 *μ*M) (b). CCK8 analysis of cell viability in OMM1 parental (OMM1-P) or OMM1 resistant (OMM1-R) cells treated with Tra with indicated concentrations for 72 h (c) or indicated times with Tra (5 *μ*M) (d). (e) Western blot detection of the phosphorylation level of ERK1/2 in OMM1-P and OMM1-R cells treated with Tra (5 *μ*M) for 24 h. (f) Quantitative analysis of p-ERK1/2 ratio to *β*-actin. (g) Western blot detection of the phosphorylation level of Akt (T308) in OMM1-P and OMM1-R cells treated with indicated concentrations of Tra for 24 h. (h) Quantitative analysis of p-Akt (T308) ratio to *β*-actin. ^∗^*P* < 0.05;  ^∗∗^*P* < 0.01;  ^∗∗∗^*P* < 0.001; two-way analysis of variance (ANOVA) in (a–d and h); one-way analysis of variance (ANOVA) in (f).

**Figure 2:** KDOAM-25 promotes cell apoptosis in MEK inhibitor-resistant UM cells. (a) CCK8 analysis of cell viability in 92.1-R cells treated with small compounds (5 *μ*M) for 72 h. O: DMSO. (b) Colony number analysis in 92.1-P and 92.1-R cells treated with KDOAM-25 (5 *μ*M) for 72 h. (c) CCK8 analysis of cell viability in 92.1-P and 92.1-R cells treated with KDOAM-25 (5 *μ*M) for 72 h. (d) FACS analysis of cell apoptosis in OMM1-P and OMM1-R cells treated with KDOAM-25 (5 *μ*M) for 24 h. (e) Quantitative analysis of percentage of cells in (d). ^∗∗^*P* < 0.01;  ^∗∗∗∗^*P* < 0.0001; one-way ANOVA in (a); two-way ANOVA in (b, c, e).

**Figure 3:** KDOAM-25 inhibits the expression of KDM5B in UM. (a) Western blot analysis of the H3K4me3 and H3K27ac in OMM1-P and OMM1-R cells treated with indicated concentrations of Tra for 24 h. (b) Quantitative analysis of H3K4me3 and H3K27ac ratio to *β*-actin. (c) Western blot analysis of the KDM5B in OMM1-P and OMM1-R cells treated with Tra (5 *μ*M) for 24 h. (d) Quantitative analysis of KDM5B ratio to *β*-actin. (e) Western blot analysis of KDM5B knockdown efficiency in OMM1-R cells. (f) Quantitative analysis of KDM5B ratio to *β*-actin. (g) The CCK8 assay of cell viability in OMM1-R cells which knockdown of KDM5B. ^∗∗^*P* < 0.01;  ^∗∗∗^*P* < 0.001;  ^∗∗∗∗^*P* < 0.0001; two-way ANOVA in (b, d, g); one-way ANOVA in (f).

**Figure 4:** KDOAM-25 directly binds to KDM5B. (a) DARTS analysis of recombinant human KDM5B proteins shows that differential pronase-mediated proteolysis after KDOAM-25 (50 *μ*M) addition is apparent for KDM5B, detected by SDS-PAGE and blotting with an *α*-KDM5B monoclonal antibody. (b) Quantitative analysis of *α*-KDM5B in (A). (C) MST analysis determined the Kd of KDOAM-25 towards His-KDM5B (487.75 nm) labeled with RED-tris-NTA 2nd Generation dye. Concentration is reported in nanomolar.

## Data Availability

We transcribed all generated data in this manuscript. For ethical and legal reasons, the individual available data could not be supplied publicly.
